The article "Hyperoxic Vasoconstriction of Human Pulmonary Arteries: A Novel Insight into Acute Ventricular Septal Defects" was published in 2013. Journal: ISRN Cardiol.

# Hyperoxic Vasoconstriction of Human Pulmonary Arteries: A Novel Insight into Acute Ventricular Septal Defects

**DOI:** 10.1155/2013/685735

**Published:** 2013-03-31

**Authors:** Priyadharshanan Ariyaratnam, Mahmoud Loubani, Robert Bennett, Steven Griffin, Mubarak A. Chaudhry, Michael E. Cowen, Levant Guvendik, Alexander R. J. Cale, Alyn H. Morice

**Affiliations:** ^1^Department of Cardiothoracic Surgery, Castle Hill Hospital, Cottingham HU16 5JQ, UK; ^2^Department of Respiratory and Cardiovascular Research, Castle Hill Hospital, Cottingham HU16 5JQ, UK

## Abstract

*Objectives*. Acute rises in pulmonary artery pressures following postinfarction ventricular septal defects present a challenge. We hypothesised that the abnormally high oxygen content exposure to the pulmonary arteries may be a factor. We investigated the contractile responses of human pulmonary arteries to changes in oxygen tension. *Methods*. Isometric tension was measured in large and medium sized pulmonary artery rings obtained from lung resections for patients with bronchial carcinoma (*n* = 30). Fresh rings were mounted in organ baths bubbled under basal conditions with hyperoxic or normoxic gas mixes and the gas tensions varied during the experiment. We studied whether voltage-gated calcium channels and nitric oxide signalling had any role in responses to oxygen changes. *Results*. Hypoxia caused a net mean relaxation of 18.1% ± 15.5 (*P* < 0.005) from hyperoxia. Subsequent hyperoxia caused a contraction of 19.2% ± 13.5 (*P* < 0.005). Arteries maintained in normoxia responded to hyperoxia with a mean constriction of 14.8% ± 3.9 (*P* < 0.005). Nifedipine inhibited the vasoconstrictive response (*P* < 0.05) whilst L-NAME had no effect on any hypoxic vasodilatory response. *Conclusions*. We demonstrate that hyperoxia leads to vasoconstriction in human pulmonary arteries. The mechanism appears to be dependent on voltage-gated calcium channels. Hyperoxic vasoconstriction may contribute to acute rises in pulmonary artery pressures.

## 1. Introduction

A postinfarction ventricular septal defect (VSD) is associated with acute rises in pulmonary artery pressures [1]. These acute rises in pulmonary artery pressure are, in turn, a significant predictor of mortality and morbidity and present a considerable challenge to the cardiac surgeon and the management of the patient in the acute intensive care setting [2].

The rise in pulmonary artery pressure may be because of failure of the right ventricle secondary to ischaemia or because of increased flow to the pulmonary artery stimulating a myogenic response. More interesting, however, is the possibility that the higher oxygen content through the pulmonary artery as a consequence of the left to right shunting of oxygenated blood may increase pulmonary artery tone especially in more subacute cases [3].

Despite lack of data on oxygen-dependent responses in *isolated* human pulmonary arteries, many potential mechanisms have been suggested in animal models. These range from calcium channel-dependent constrictive pathways to vasodilatory pathways involving Nitric Oxide (NO) release by the endothelium [4, 5]. 

Here we sought to evaluate the differential effect of hypoxia and subsequent reoxygenation on the vascular tone in isolated human pulmonary arteries invitro. We used a selective blocker (nifedipine) of L-type voltage-gated calcium channels and a selective blocker (L-NAME) of endothelial nitric oxide Synthase to elucidate their involvement in the responses to changes in oxygen tension. 

## 2. Methods

### 2.1. Study Model and Design

Informed consent was obtained for human lung tissue obtained from patients undergoing surgery for bronchial carcinoma at Castle Hill Hospital, Cottingham, UK. Ethical approval for this project was obtained from the Regional Ethics Committee.

 Extralobar (mean internal diameter 4 mm) and medium sized intralobar (mean internal diameter 2 mm) pulmonary arteries were dissected from healthy areas of lung resections (*n* = 30). Arteries were cut into 5 mm thickness rings.

Vessels were mounted between stainless steel wires connected to an isometric force transducer (Dynamometer UFI Devices, UK). The rings were immersed in a 25 mL water jacketed organ bath (Radnoti, USA) containing Krebs-Henseleit (Krebs) solution warmed to 37°C. Oxygen was bubbled at varying concentrations (0% hypoxia, 21% normoxia, and 95% hyperoxia, balance N_2_) and CO_2_ was kept constant at 5% to maintain a pH of 7.4.

### 2.2. Experimental Protocols

A resting tension of 1-2 g was applied and the vessels were allowed to equilibrate for 60 minutes. The endothelial integrity of each vessel was confirmed by significant vasodilatation to acetylcholine (ACh, 1 mM) before the experimental protocol. Smooth muscle viability was confirmed by exposure to potassium chloride (30 mM KCl) at the end of the experiment. Any arteries not responding to KCl were excluded from the analysis. 

#### 2.2.1. Effect of H-R on Vessels Maintained in 95% O_2_

 Vessels (*n* = 13) were equilibrated for 60 minutes in *hyperoxic *conditions and resting tension was recorded. Vessels were then exposed to 30 minutes of hypoxia and subsequently reoxygenated with hyperoxia for 30 minutes and tension was recorded. 

#### 2.2.2. Effect of H-R on Vessels Maintained in 21% O_2_

Vessels (*n* = 6) were left to equilibrate for 1 hour in *normoxic* conditions and resting tension was recorded. Vessels were then exposed to 20 minutes of hypoxia and subsequently reoxygenated with hyperoxia for 30 minutes and tension was recorded.

#### 2.2.3. Effect of Calcium L-Type Channels on the Vasoconstrictive Response

Vessels (*n* = 6) were left to equilibrate for 1 hour in *hyperoxic* conditions and resting tension was recorded. Vessels were then exposed to 30 minutes of hypoxia. Nifedipine (5 *μ*M) was added and arteries were reoxygenated with hyperoxia for 30 minutes.

#### 2.2.4. Effect of L-NAME on Hypoxia-Reoxygenation

Vessels (*n* = 5) were left to equilibrate for 1 hour in *hyperoxic* conditions and resting tension was recorded. Vessels were then exposed to 30 minutes of hypoxia and subsequently reoxygenated with hyperoxia for 30 minutes and tension was recorded. L-NAME (1 mM) was added and hypoxia-reoxygenation was repeated.

*Reagents Used.* Krebs bicarbonate solution consisted of 113.8 mM NaCl, 4.7 mM KCl, 1.2 mM MgSO_4_, 25 mM NaHCO_3_, 1.2 mM KH_2_PO_4_, 11.4 mM glucose, and 2.4 mM CaCl_2_ dissolved in deionised water. Reagents were from Fisher Scientific (UK) except Nifedipine (Tocris, USA), L-NAME (Tocris, USA), and acetylcholine chloride (Sigma-Aldrich, UK). Gas mixtures were from the Linde Group (UK). Oxygen saturations in the organ baths were measured using an oxygen probe (ArrowLab).

### 2.3. Analysis of Data

Tensions were recorded on Lab Chart (ADInstruments, UK). Contractions or dilations of pulmonary artery are expressed as a percentage of the maximal contraction to 30 mM KCl (KCl max). Data are presented as means ± standard deviation. Statistical analysis was carried out by paired Student's *t*-tests for repeated measurement analyses.

## 3. Results

### 3.1. Effect of H-R on Vessels Resting in 95% O_2_

All vessels dilated in response to hypoxia. The mean vasodilatory response was 18.1% ±15.6 (*P* < 0.005). Upon reoxygenation vessels responded with a mean vasoconstriction of 19.2% ±13.5 (*P* < 0.005). Thus, vessels did not constrict above their resting tension (Figure 1). 

### 3.2. Effect of H-R on Vessels Resting in 21% O_2_

In vessels maintained in normoxia, there was no significant vasodilatory effect of hypoxia (*P* > 0.05). However, vessels constricted in response to subsequent hyperoxia with a net mean vasoconstriction of 14.8% (±3.9, *P* < 0.005) above RT.

### 3.3. Effect of Nifedipine on H-R

Nifedipine blocked the vasoconstrictive effects of hyperoxia (*P* < 0.05) (Figure 2).

### 3.4. Effect of L-NAME on Responses to Hypoxia

Arteries dilated significantly (*P* < 0.05) to hypoxia. However, there was no significant difference (*P* > 0.05) in dilation in response to hypoxia in the absence or presence of L-NAME (30.5% ±21.9 versus 42.0 ± 17.5, resp.) (Figure 3).

### 3.5. Effect of Vessel Size on Hypoxia-Reoxygenation

There was no significant difference (*P* > 0.05) in any of the protocols regarding the effect of vessel size on the response to hypoxia-reoxygenation.

## 4. Discussion

To date, the vast majority of data concerning the effects of oxygen on pulmonary arteries have been restricted to animal models. The main reason for this is likely to be the difficulty of obtaining pulmonary artery tissue from patients. Whilst studies have evaluated the effects of oxygen on isolated pulmonary artery smooth muscle cells, little data exists on the synergy of these cells within arterial rings or perfused lung models.

We used medium and large pulmonary artery rings for two reasons. Firstly, these can be more easily obtained from lobectomy samples than small resistance arteries without affecting tumour staging and analysis. Secondly, studies have shown that it is these arteries which largely determine pulmonary vascular tone and the subsequent strain on the right heart [6, 7]. 

 Our human study consistently shows that hyperoxia causes vasoconstriction. We believe that this represents a return to a greater basal tone in hyperoxic conditions since arteries *originally maintained in normoxia* prior to hypoxic challenge demonstrated a net vasoconstriction above their basal tone. 

Vasoconstrictive responses to oxygen in animal models have invariably been associated with calcium. However, the source of this calcium remains uncertain as both release from intracellular stores and influx from the extracellular compartment have been implicated [8]. Our results in human arteries demonstrate that this response is dependent on L-type voltage-gated calcium channels as demonstrated by the lack of any hyperoxic vasoconstriction in the presence of nifedipine. 

In our pulmonary arteries we consistently show that L-NAME does not affect the dilation induced by hypoxia. NO is produced by the endothelium by endothelial NO synthase (eNOS) which is blocked by L-NAME. This indicates that the hypoxic vasodilatation is independent of an NO-mediated effect on pulmonary artery smooth muscle. The majority, but not all arteries, responded to acetylcholine. Hence we cannot exclude the fact that the endothelium may have been denuded upon harvesting the pulmonary artery from the lobectomy specimen. However, as acetylcholine unresponsive arteries still dilated to hypoxia, it appears that the endothelium does not play a significant role in the vasoactive responses to either hypoxia or hyperoxia.

Human pulmonary arteries are normally exposed to hypoxic conditions. The normal partial pressures of oxygen in the human pulmonary artery range from 2 to 6 KPa which are similar to those when our arteries are maintained in 0% O_2_. Patients with acute post infarction VSDs often necessitate a high oxygen delivery to the lungs in the resuscitative phase. This high oxygen delivery across the VSD to the pulmonary artery ranges between 40 KPa and 60 KPa which is similar to that produced in our Krebs solution when arteries are exposed to 95% O_2_. 

By removing hyperaemic factors and contributions of perfusion pressure and by studying rings in isolation, our results indicate that there may be an element of hyperoxic vasoconstriction contributing to the raised pulmonary artery pressures following acute VSDs.

*Limitations and Future Work*. Our results may be due to an isolated “in vitro artifact.” One can speculate that the effect would be different in perfused lung model, and we agree that perfused models would need to be undertaken to confirm this isolated artery phenomenon, preferably with blood medium rather than the asanguineous medium of Krebs. Further to this, we used pulmonary arteries from lung cancer patients. Although there was no recorded evidence of pulmonary hypertension or pulmonary vascular disease preoperatively, it would be prudent to investigate whether this phenomenon extends to those people without lung cancer.

## 5. Conclusions

Our study is the first to demonstrate that hyperoxic vasoconstriction in large and medium sized human pulmonary arteries is dependent upon voltage-gated calcium channels. This mechanism may contribute to the acute rises in pulmonary artery pressures following post infarction VSDs. It provides an avenue of further investigation to pursue potential targets of pulmonary hypertension in the acute cardiac surgical patients. 

## Figures and Tables

**Figure 1:** Response of arteries to H-R resting in 95% O_2_.

**Figure 2:** Effect of Nifedipine on the vasoconstrictive response to hyperoxia.

**Figure 3:** Effect of L-NAME on the vasodilatory response to hypoxia.

## Abbreviations

Ach: Acetylcholine
H-R: Hypoxia-reoxygenation
KCl: Potassium chloride
L-NAME: N-nitro-L-arginine methyl ester
NO: Nitric oxide.

## References

[1] Coskun KO, Coskun ST, Popov AF (2009). Experiences with surgical treatment of ventricle septal defect as a post infarction complication. *Journal of Cardiothoracic Surgery*.

[2] Denault A, Deschamps A, Tardif JC, Lambert J, Perrault L (2010). Pulmonary hypertension in cardiac surgery. *Current Cardiology Reviews*.

[3] Corno AF, Tozzi P, Genton CY, Von Segesser LK (2003). Surgically induced unilateral pulmonary hypertension: time-related analysis of a new experimental model. *European Journal of Cardio-Thoracic Surgery*.

[4] Norton CE, Jernigan NL, Kanagy NL, Walker BR, Resta TC (2011). Intermittent hypoxia augments pulmonary vascular smooth muscle reactivity to NO: regulation by reactive oxygen species. *Journal of Applied Physiology*.

[5] Weir EK, Olschewski A (2006). Role of ion channels in acute and chronic responses of the pulmonary vasculature to hypoxia. *Cardiovascular Research*.

[6] Gan CTJ, Lankhaar JW, Westerhof N (2007). Noninvasively assessed pulmonary artery stiffness predicts mortality in pulmonary arterial hypertension. *Chest*.

[7] Mahapatra S, Nishimura RA, Oh JK, McGoon MD (2006). The prognostic value of pulmonary vascular capacitance determined by Doppler echocardiography in patients with pulmonary arterial hypertension. *Journal of the American Society of Echocardiography*.

[8] Ward JPT, Snetkov VA, Aaronson PI (2004). Calcium, mitochondria and oxygen sensing in the pulmonary circulation. *Cell Calcium*.

